# Fbxw7 and Skp2 Regulate Stem Cell Switch between Quiescence and Mitotic Division in Lung Adenocarcinoma

**DOI:** 10.1155/2019/9648269

**Published:** 2019-08-25

**Authors:** Wenzhu Zhang, Zihan Ren, Lanling Jia, Xin Li, Xinshan Jia, Yuchen Han

**Affiliations:** ^1^Department of Pathology, College of Basic Medical Sciences, China Medical University, Shenyang, China; ^2^Department of Pathology, The First Affiliated Hospital of China Medical University, Shenyang, China; ^3^Department of Otorhinolaryngology, The First Affiliated Hospital of China Medical University, Shenyang, China; ^4^Department of Physiology, College of Life Science and Biopharmaceutics of Shenyang Pharmaceutical University, Shenyang, China

## Abstract

**Background/Aims:**

The molecular mechanism of dormancy initiation of cancer stem cells (CSCs) is not clear. This study was to explore the molecular mechanism by which CSCs switch from mitotic division to quiescence.

**Methods:**

MTT assays, flow cytometry, Western blotting, qRT-PCR, and immunofluorescence staining were used to test cell viability, cell cycle and expression of* F*-box and WD repeat domain-containing 7 (Fbxw7),* c*-myc, S phase kinase associated protein-2 (Skp2), cyclin-dependent kinase inhibitor 1B (p27), octamer-binding transcription factor 3/4 (Oct3/4), and *β* catenin gene in 5-fluorouracil (5-FU)-treated A549 cells. Lung adenocarcinoma xenograft models were employed to detect the effects of Fbxw7 on tumor growth.

**Results:**

5-FU inhibited the proliferation of A549 cells, with a median inhibitory concentration (IC50) of 200 *μ*g/ml after 24 h treatment. 5-FU treatment increased the expressions of Oct3/4, Fbxw7, and p27 and increased the number of A549 cells at G0/G1. 5-FU treatment triggered nuclear translocation of *β*-catenin, decreased the expression levels of c-myc and Skp2, and decreased the number of A549 cells at S phase. Release from 5-FU decreased the expressions of Oct3/4, Fbxw7 and p27; decreased the percentage of cells in the G0/G1 phase; increased the expressions of Skp2 and c-myc; and increased the proportion of cells in S phase. 5-FU treatment led to high expressions of Oct3/4, c-myc, and p27, with low expressions of Fbxw7 and Skp2. Knockdown of Fbxw7 augmented the expression of c-myc and decreased the proportion of A549 cells in Go/G1 phase. Skp2 siRNA increased the expression of p27 and the percentage of G0/G1 phase cells and reduced the proportion of S phase cells. Fbxw7 overexpression inhibited tumor growth in mouse lung adenocarcinoma xenograft models. When Fbxw7 expression was low, Skp2 expression was higher in lung adenocarcinoma tissues and associated with the differentiation of lung adenocarcinoma.

**Conclusion:**

5-FU enriches the CSCs in lung adenocarcinoma cells* via* increasing Fbxw7 and decreasing Skp2 expression, followed by downregulation of c-myc and upregulation of p27, which switches cells to quiescence.

## 1. Introduction

Lung cancer is one of the most common malignant tumors worldwide and the leading cause of cancer death in China [1]. The majority (80%) of lung cancer is non-small-cell lung cancer (NSCLC), among which adenocarcinoma is the most common histological type comprising 30-50% of NSCLC cases [2, 3]. Although great advances have been made in lung cancer therapy, metastasis and recurrence of lung cancer often result in high mortality and novel targeted chemo- and radiotherapies are urgently desired [4–6]. Cancer stem cells (CSCs) have been identified in a variety of cancers including lung cancer. The characteristics of CSCs are cell quiescence, where cells are not dividing and arrested in the G0/G1 phase of the cell cycle [7, 8], pluripotency and self-renewal properties [9, 10], and production of a heterogeneous population of tumor cells [9, 10]. CSCs appear to have lower proliferation rates and higher expression of DNA repair and antiapoptotic genes than normal cells, which can result in treatment failure [11]. Genes in CSCs, such as* Oct4*,* Nanog*,* nestin*, and* cytokeratin 19* (*CK19*), are upregulated, while* involucrin *and* CK13* are downregulated. Adult stem cells in the body are generally in a state of dormancy or the G0 phase of the cell cycle. Stem cells can be activated to reenter the cell cycle* via* stimulation by specific environmental or internal factors [12]. Deregulation of CSC dormancy in lung adenocarcinoma contributes to the generation of leukemia stem cells, leading to cancer metastasis and recurrence [13]. At present, studies on stem cell activation and dormancy mainly focus on hematopoietic cells, melanocytes, epidermal cells, and CSCs [12, 14]. It has been proposed that phosphorylation of RNA polymerase,* p27* gene regulation, autophagy, biochronometer theory, and regulation of the TGF-*β*/Smad pathway and the insulin/IGF1 pathway are mechanisms of the underlying dormancy and activation of stem cells [12, 14]. Lung CSCs have the abilities to self-renew, differentiate, and proliferate. They are highly resistant to chemotherapy, and can give rise to tumor cells during cancer development, resulting in cancer metastasis, recurrence [13, 15], and failure of therapy [7, 8].

The antimetabolite drug 5-fluorouracil (5-FU) is widely used in the treatment of numerous cancers, including lung cancer. It induces cell cycle arrest and apoptosis, and inhibits the proliferation of cells in the S phase [16]. Unfortunately, most cancer patients develop resistance to 5-FU. 5-FU was reported to be associated with cancer stem cell enrichment, enhancing stemlike traits in colon cancer cells [17], augmenting expression of stem cell markers like octamer-binding transcription factor 4 (Oct4) Oct4 and CD133, decreasing the expression of differentiation markers like CD24 [18–21], increasing the percentage of side population (SP) cells in lung adenocarcinoma cell line SPC-A1 [21], and increasing the ability to form colonies [18–20].

However, the molecular mechanism of 5-FU enrichment of lung adenocarcinoma stem cells and its effects on dormancy initiation of stem cells are not yet clear. Enhancing our understanding of the molecular mechanisms of CSC dormancy may promote the development of 5FU therapy and improve the overall prognosis of patients with lung adenocarcinoma.

*F*-box and WD repeat domain-containing 7 (Fbxw7) and S phase kinase associated protein-2 (Skp2) are both* F*-box proteins that are responsible for substrate recognition by an SCF (Skp1Cul1-F-box protein)-type E3 ubiquitin ligase complex. The* Fbxw7* gene participates in ubiquitination and degradation of targeted oncogenes [22, 23]. Fbxw7 is frequently mutated in many human malignancies, and low Fbxw7 expression is correlated with stem cell renewal and EMT [24–27]. On the contrary, Skp2 has been reported to interact with multiple signaling pathways including Akt and pRb, and genetic silencing of Skp2 restricted the development of tumors driven by these pathway alterations [28, 29]. The clinical observations also indicate that Fbxw7 is crucial for preventing carcinogenesis as a result of its role in cell cycle regulation, and Skp2 is overexpressed in prostate cancer and its overexpression is correlated with tumor stage, recurrence and poor patient survival [30, 31]. Thus, enhanced Fbxw7 expression and declined Skp2 expression may be involved in the switch of CSCs between quiescence and active cell division.

In this study, the mechanism underlying 5-FU treatment induced CSC enrichment was explored using gene knockdown strategy. It was demonstrated that Fbxw7 contributed to 5-FU treatment induced CSC quiescence while Skp2 enhanced CSC division. Our results indicate that Fbxw7 and Skp2 may be potential therapeutic targets of lung adenocarcinoma.

## 2. Materials and Methods

### 2.1. Clinical Specimens and Cell Culture

Forty paired lung adenocarcinoma and corresponding normal tissue samples were collected at Department of Pathology of the First Affiliated Hospital of China Medical University, after written consent was obtained from all patients. All tissue samples were stored at −80°C until use. Lung adenocarcinoma cell line A549 was obtained from Shanghai Institute of Biochemistry and Cell Biology, Chinese Academy of Medical Sciences (Shanghai, China). A549 cells were cultured in RPMI-1640 (Hyclone, USA) containing 10% (v/v) fetal bovine serum (FBS, Hyclone, USA), 2 mM Gln, 100 units/ml penicillin, and 100 *μ*g/mL streptomycin, in a humidified incubator (5% CO_2_ in air) at 37°C.

### 2.2. MTT Assays

The cytotoxicity of 5-FU was determined by using 3-(4,5-dimethylthiazol-2-yl)-2,5-diphenyl tetrazolium bromide (MTT) assays. A549 cells were cultured on 96-well plates with 100 *μ*L of growth medium. After treatment with 5-FU at concentrations of 10 *μ*g/mL, 25 *μ*g/mL, 50 *μ*g/mL, 100 *μ*g/mL, 200 *μ*g/mL, 400 *μ*g/mL, 800 *μ*g/mL or 1000 *μ*g/mL for different hours (24 h, 48 h or 72 h), the media were replenished and 10 *μ*L MTT dye (5 mg/mL) was added. After 4 h incubation at 37°C, the MTT solution was replaced with 150 *μ*L of DMSO. Optical density was measured at 490 nm using a microplate reader (Sunrise RC, Tecan, Switzerland). The half maximal inhibitory concentration (IC50) was calculated as the drug concentration required to reduce cell survival by 50%. The A549 cells were then divided into 3 groups: the control group (N), cells treated with 200 *μ*g/ml 5-FU for 24 h (the 0 h group), and cells treated with 200 *μ*g/mL 5FU for 24 h followed by culturing in the media without 5-FU for 48 h (the 48 h group). Cells were collected for the corresponding analysis.

### 2.3. Immunofluorescence Microscopy

Immunofluorescence was performed as described previously [32]. Cells were fixed in 4% paraformaldehyde in 20 mM HEPES (pH 7.4) for 20 min, washed three times, and permeabilized with 1.0% Triton X-100 for 5 min. Cells were then incubated with rabbit polyclonal anti-Oct4 antibody (1:200, Santa Cruz Biotechnology, Santa Cruz, CA, USA), mouse polyclonal anti-*β* catenin antibody (1:200, Santa Cruz Biotechnology), mouse polyclonal anti-Fbxw7 antibody (1:200, Santa Cruz Biotechnology), mouse polyclonal antic-myc antibody (1:200, Santa Cruz Biotechnology), mouse polyclonal anti-Skp2 antibody (1:200, Santa Cruz Biotechnology) or mouse polyclonal anti-p27 antibody (1:200, Santa Cruz Biotechnology) overnight at 4°C before being washed three times and incubated with goat anti-rabbit conjugated secondary antibody or goat anti-mouse conjugated secondary antibody correspondingly for 1 h at room temperature in the dark. DAPI was used for nuclear counterstaining. The stained cells were mounted and viewed under a BX51 inverted epifluorescence microscope (Olympus, Tokyo, Japan).

### 2.4. Cell Cycle Analysis

Totally 10^6^ cells were plated in each well of a six-well plate. The cells in three wells were treated with 200 *μ*g/mL 5-FU; the cells in the other three wells were used as control. After 24 h treatment, cells were fixed overnight at 4°C with 70% ethanol. The number of cells at different phases of cell cycle was analyzed by measuring DNA fragment staining with propidium iodide (PI) using flow cytometry.

### 2.5. Small Interfering RNA Transfection

Human Fbxw7 and Skp2 siRNA were produced by Reibo Co. Ltd (Guangzhou, China). The sequences of human siRNAs were as follows: si-Fbxw7, 5′-ACAGGACAGUGUUUACAAA-3′; siSkp2, 5′-UCUUAGCGGCUACAGAAAG-3′. Briefly, cells were transfected with the small interfering RNA using oligofectamine (Invitrogen) according to the manufacturer's instruction.

### 2.6. RNA Extraction and Quantitative RT-PCR (qRT-PCR)

Total RNA was extracted from the cells using TRIzol® reagent, and cDNA was synthesized using M-MLV-RT and Oligo-dT primers (Promega, USA) in 20 *μ*L RT buffer. Real-time PCR was performed using the SYBR Premix Ex Tag Kit (TaKaRa, Japan) in an ABI 7300 Sequencing Detection System (Applied Biosystems, Foster City, CA, USA). The PCR was run for 1 cycle, 95°C, 10 min; 35 cycles, 95°C for 10s, 60°C for15s; and 1 cycle, 72°C for 10 s. The sequences of the oligonucleotide primers are shown as Table 1.

### 2.7. Western Blotting Analysis

Cells were harvested and lysed in the RIPA buffer (Sigma-Aldrich, USA). Protein concentrations were determined using the BCA protein assay kit (Thermo Fisher Scientific, USA). Proteins (30 *μ*g) were separated by 10% SDS-PAGE and transferred onto a nitrocellulose membrane. After being blocked with BSA, the membranes were then incubated with primary antibodies against Fbxw7, Skp2, OCT4, c-myc, p27 (Santa Cruz Biotechnology) and GAPDH (Santa Cruz Biotechnology), respectively, at 4°C overnight. After being washed three times for 15 min with TBST solution, the membrane was further incubated with appropriate HRP conjugated secondary antibodies in PBS-T solution for 2 h at room temperature. The membrane was washed three times for 15 min in TBST solution and incubated with ECL solution for 1 min. Signals were detected using the ECL chemiluminescence method. Relative protein levels were quantified using GAPDH as internal standard reference.

### 2.8. Nude Mouse Xenograft Experiments

The animal experiments were approved by the Ethics Committees of China Medical University. Six week old male BALB/c nude (nu/nu) mice were purchased from the Department of Laboratory Animal Science of China Medical University (n=10). Nude mice were maintained in a specific pathogen-free animal facility and all animal experiments were performed in accordance with the regulations of the Institutional Animal Care and Use Committee (IACUC). Nude mice (National Rodent Laboratory Animal Resource) between 5-6 weeks of age were subcutaneously injected with 3 × 10^5^ A549 cells or Fbxw7-overexpressing A549 cells. Animals were sacrificed 26 days after injection of tumor cells, and tumors were weighed.

### 2.9. Immunohistochemistry

Immunohistochemical staining was performed as described by Li [33] with minor modification. Human lung adenocarcinoma tissues and normal tissues were paraffin embedded, and 4 *μ*m sections were prepared. Paraffin sections were dewaxed in xylene and rehydrated in gradient alcohols. Antigen retrieval was performed by heating the sections for 1.5 min in 0.01 M citrate buffer, pH 6.0. Nonspecific staining was reduced by incubation in blocking buffer containing goat serum (SP KIT-B1; Maixin-Bio, Fuzhou, China) for 30 min. Then, the sections were incubated with Fbxw7 and Skp2 antibody (Santa Cruz Biotechnology) overnight at 4°C, followed by incubation with appropriate secondary antibodies for 30 min. The reaction was visualized using DAB (DAB-0031; Maixin-Bio) plus chromogen. Specimens were examined using a BX51 microscope (Olympus). Sections treated with 1% BSA in PBS instead of the primary antibody were used as a negative control.

### 2.10. Statistical Analysis

Statistical analysis was carried out using SPSS version 19.0 (IBM Chicago, IL, USA). All tests were performed in triplicate and presented as mean ± SD. Comparisons between two groups were tested using Student's *t* test (two tailed). One-way analysis of variance (ANOVA) followed by Tukey* post hoc* test was used for multiple comparison. P<0.05 was considered statistically significant.

## 3. Results

### 3.1. Effects of 5-FU on Lung Adenocarcinoma Cell Line A549 Cells

5-FU inhibited the proliferation of A549 cells in a time- and dose-dependent manner (Figure 1(a)).

The median IC50 of 5-FU for 24 h was 200 *μ*g/ml, which was chosen as the dose for subsequent experiments. 5-FU treatment significantly (p<0.05) increased the protein and mRNA levels of a stem cell marker Oct3/4, while the upregulation of Oct3/4 expression was significantly reversed after 5-FU was removed for 48 h (Figures 1(b) and 1(c)). Immunofluorescence assay revealed that 5-FU treatment significantly augmented Oct3/4 expression (Figure 1(d)), and triggered a significant nuclear translocation of *β*-catenin in A549 cells (Figure 1(e)).

The number of A549 cells at S phase significantly decreased (22.02 ± 0.69% vs. 7.8 ± 1.78%, *p* < 0.05) and the number of A549 cells at G0/G1 phase significantly increased (69.64 ± 0.34% vs. 88.98 ± 1.78%, *p* < 0.05) after A549 cells were treated with 5-FU for 24 h (Figures 1(f) and 1(g)). In contrast, the proportion of cells in S phase was dramatically increased, and the percentage of cells in the G0/G1 phase decreased (Figures 1(f) and 1(g)), after 5-FU treated A549 cells were released from 5-FU and cultured in routine media for 48 h.

### 3.2. Effects of 5-FU on the Expression of Fbxw7, p27, Skp2, and c-myc

5-FU treatment significantly (p < 0.05) increased the protein levels of Fbxw7 and p27, and decreased the protein levels of c-myc and Skp2 (Figure 2(a)). In contrast, the protein levels of Fbxw7 and p27 significantly decreased, and the protein levels of Skp2 and c-myc increased, after 5-FU treated A549 cells were released from 5-FU and cultured in routine media for 48 h (Figure 2(a)). 5FU increased the mRNA levels of Fbxw7 and p27, and decreased the mRNA levels of Skp2 and c-Myc (Figure 2(b)).

### 3.3. Coexpression of Oct3/4, Fbxw7, c-myc, Skp2, and p27 in 5-FU Treated A549 Cells

The coexpression of Oct3/4, Fbxw7, c-myc, Skp2, and p27 in 5-FU treated A549 cells was detected using immunofluorescence assay with antibodies against Oct3/4, Fbxw7, c-Myc, Skp2, and p27. In untreated A549 cells, Oct3/4 was negative, while Fbxw7 was positive and the downstream protein c-myc was negative (Figures 3(a) and 3(b)). After cells were exposed to 5-FU, the expression of Oct3/4 was increased, Fbxw7 and Skp2 declined, and c-myc and p27 were highly expressed (Figures 3(c) and 3(d)).

### 3.4. Effects of Knockdown of Fbxw7 and Skp2 on Cell Cycle and the Expression of c-myc and p27

Knockdown of Fbxw7 significantly augmented the protein and mRNA expression levels of c-myc (Figures 4(a) and 4(b)). Similarly, Skp2 siRNA increased the protein and mRNA levels of p27 (Figures 4(c) and 4(d)). Knockdown of Fbxw7 significantly decreased the proportion of cells in Go/G1 phase in A549 cells (Figure 4(e)). On the contrary, knockdown of Skp2 increased the percentage of cells in the G0/G1 phase and reduced the proportion of cells in the S phase.

### 3.5. Effects of Fbxw7 on Tumor Growth in Mouse Lung Adenocarcinoma Xenograft Models

Mice injected with untreated A549 cells had tumors with an average volume of 1500 mm^3^, whereas little tumor growth was observed in mice injected with Fbxw7-overexpressing A549 cells (Figures 5(a) and 5(b)). Fbxw7 overexpression significantly (p<0.05) decreased the tumor weight compared with control group (Figure 5(c)). Hematoxylin and eosin (H&E) staining showed that Fbxw7 decreased tumor growth* in vivo*, resulting in cells with smaller nuclei and slightly atypical cells occasionally having two nuclei (Figure 5(d)). Altogether, these results showed that Fbxw7 inhibited tumor growth in A549 lung adenocarcinoma xenograft models

### 3.6. Expression of Fbxw7 and Skp2 in Lung Adenocarcinoma Tissues

Immunohistochemistry revealed that the poorly differentiated cancer tissues were Fbxw7 positive in fewer than 40% of 40 lung adenocarcinoma patients, while 80% of the adjacent nontumor tissues were Fbxw7 positive (Figures 6(a) and 6(b)). In addition, Skp2 was positively expressed in the lung adenocarcinoma tissues and associated with the differentiation of lung adenocarcinoma (Figures 6(c) and 6(d)).

## 4. Discussion

In this study, 5-FU was found to enrich the CSC population in lung adenocarcinoma. Cell biology, molecular biology and immunofluorescence analysis demonstrated that 5-FU enriched the CSCs through modulating the Fbxw7-c-myc axis by increasing Fbxw7 expression, decreasing c-myc expression, and switching cells to quiescence, and modulating the Skp2-p27 axis by decreasing Skp2 expression, increasing p27 expression, and switching cells to active division.

It was found that 5-FU inhibited the proliferation, increased the protein and mRNA levels of a stem cell marker Oct3/4 and triggered a significant nuclear translocation of *β*-catenin, in A549 cells. 5-FU also decreased the number of A549 cells at S phase, increased the number of A549 cells at G0/G1, whereas release of A549 cells from treatment of 5-FU decreased Oct3/4 expression, increased the proportion of cells in S phase, and decreased the percentage of cells in the G0/G1 phase. These findings are consistent with the previous observations that 5-FU enhanced stemlike traits [33], increasing expression of stem cell markers and percentage of SP cells in lung adenocarcinoma cell line SPC-A1 [33, 34]. These results demonstrated that 5-FU enriched CSC population in lung adenocarcinoma cells [34].

Fbxw7 was identified as a tumor suppressor gene that participated in ubiquitination and degradation of oncogenes [22, 23, 35], including c-myc, which is supported by our observation that knockdown of Fbxw7 augmented the protein and mRNA expression levels of c-myc.* c‐myc *is a proto‐oncogene and is activated in over half of human cancers [36]. 5FU treatment caused an increase in Fbxw7 expression and a decrease in c-myc expression. The release of 5-FU led to a decrease in the protein level of Fbxw7 and an increase in the protein level of c-myc. Together, the data suggests that there is a regulatory relationship between 5-FU and the Fbxw7-c-myc axis. The coexistence of negative Oct3/4 with a low expression of Fbxw7 and high expression of c-myc in untreated A549 cells, and the coexistence of a higher expression of Oct3/4 with a high expression of Fbxw7 and low expression of c-myc in 5-FU treated cells indicate that the Fbxw7-c-myc axis is involved in modulating CSC enrichment[24]. Consistent with the previous observation [25], Fbxw7 had a lower expression level in lung adenocarcinoma tissues than the adjacent nontumor tissues. Knockdown of Fbxw7 augmented the protein and mRNA expression levels of c-myc, and decreased the proportion of A549cells in the Go/G1 phase. Fbxw7 overexpression reduced tumor growth and decreased tumor weight in mouse lung adenocarcinoma xenograft models. All these results indicate that 5-FU enriched CSCs through modulating the Fbxw7-c-myc axis by increasing Fbxw7 expression, decreasing c-myc expression, arresting cells at the Go/G1 phase, and suppressing tumor growth. Skp2 is a component of the E3 ubiquitin ligase, which promotes the ubiquitination-associated degradation of a cyclin-dependent kinase inhibitor p27, and increases NSCLC growth [37, 38]. Under physiological conditions, Skp2 controls the initiation of mitosis in that its expression peaks at the S and G2 phases, but not G0 and G1 phase [37, 38]. 5-FU mediated a decrease in Skp2 expression and increase in p27 expression, and the release of 5-FU mediated an increase in Skp2 expression and decrease in p27 expression, suggesting that there is a regulatory relationship between 5-FU and the Skp2-p27 axis [37, 38]. The coexistence of a negative Oct3/4 with a high expression of Skp2 and low expression of p27 in untreated cells, and the coexistence of a higher expression of Oct3/4 with decreased expression of Skp2 and high expression of p27 in 5-FU treated cells suggest that the Skp2-p27 axis involved in CSC enrichment. Skp2 siRNA increased the protein and mRNA levels of p27, increased the percentage of G0/G1 phase cells, and reduced the proportion of S phase cells. Skp2 was highly expressed in lung adenocarcinoma tissues and associated with differentiation of lung adenocarcinoma, which was also observed in previous studies [26, 39–43]. All these results demonstrated that 5-FU enriched CSCs through modulating the Skp2-p27 axis by decreasing Skp2 expression, increasing p27 expression, and switching cells to quiescence.

In conclusion, Fbxw7 promotes CSCs to switch to quiescence, and Skp3 promotes CSCs to switch to active mitotic division. Fbxw7 exerts a potent inhibitory effect on A549 tumor growth* in vivo* and is associated with decreased clinical progression of lung adenocarcinoma. 5-FU enriches CSCs in lung adenocarcinoma cells* via* increasing Fbxw7 and decreasing Skp2 expression, followed by downregulation of c-myc, upregulation of p27, and switching cells to quiescence. Our findings suggest that Fbxw7 and Skp2 may be potent therapeutic targets for intervening the switch of CSCs between quiescence and active mitotic division in lung adenocarcinoma and relieving CSCs-mediated drug-resistance.

## Figures and Tables

**Figure 1:** Influence of 5-Fu on A549 cells. (a) Survival rates of A549 cells exposed to 5-Fu for 24 h, 48 h, or 72 h. Cell viability was detected by the MTT assay. (b) The protein expression of OCT4 in the N group, 0 h group, and 48 h group was determined by Western blotting assays. (c) The mRNA expression of OCT4 in the N group, 0 h group, and 48 h group was determined by qRT-PCR. (d) Effect of 5-Fu treatment on OCT4 protein expression was assessed by immunofluorescence microscopy. (e) The expression of *β*-catenin in A549 cells with or without 5-Fu treatment. (f) Effect of 5-Fu treatment and release of 5-Fu treatment for 48 h on A549 cell cycle distribution. Cell cycle distribution of G0/G1 and S phases was measured by flow cytometry. (g) The percentage of cells at different cycle phases was calculated. All the results are expressed as mean ± SD (n = 3, *∗* p < 0.05 significantly different from control group).

**Figure 2:** Expression of Fbxw7, p27, Skp2, and c-myc in 5-Fu treated A549 cells. (a) Comparison of the protein expression of Fbxw7, c-myc, Skp2, and p27 among the control A549 cells, A549 cells treated with 5-Fu for 24 h, and A549 cells released from 5-Fu for 48 h. (b) Comparison of the mRNA expression of Fbxw7, c-myc, Skp2, and p27 among the control A549 cells, A549 cells treated with 5-Fu for 24 h, and A549 cells released from 5-Fu for 48 h. All the results are expressed as mean ± SD (n = 3, *∗* p < 0.05 significantly different from control group).

**Figure 3:** Coexistence of Oct4/3, the Fbxw7/c-myc axis, and the Skp2-p27 axis in 5-Fu treated A549 cells. (a) Costaining of Fbxw7 and Oct4 was detected by immunofluorescence microscopy with or without 5-Fu treatment. (b) Costaining of c-myc and Oct4 was detected by immunofluorescence microscopy with or without microscopy assay with or without 5-Fu treatment. (d) Costaining of p27 and Oct4 was detected by immunofluorescence microscopy with or without 5-Fu treatment.

**Figure 4:** Effects of Fbxw7 and Skp2 on the cell cycle and the expression of c-myc and p27. (a) The protein expression of c-myc was determined by Western blotting assays in A549 cells after transfection with Fbxw7 siRNA. (a) The mRNA expression of c-myc was determined by qRT-PCR in A549 cells after transfection with Fbxw7 siRNA. (c) The protein expression of p27 was determined by Western blotting assays in A549 cells after transfection with Skp2 siRNA. (d) The mRNA expression of p27 was determined by qRT-PCR in A549 cells after transfection with Skp2 siRNA. (e) Effects of the Fbxw7 siRNA and Skp2 siRNA on A549 cell cycle distribution. Cell cycle distribution of G0/G1 and S phases was measured by flow cytometry. (f) The percentage of cells at different cycle phases was calculated. All the results are shown as mean ± SD (n = 3, *∗* p < 0.05, significantly different from control group).

**Figure 5:** Fbxw7 inhibits tumor growth in lung adenocarcinoma xenograft models. (a) 3 × 10^5^ A549 cells and 3 × 10^5^ A549 cells with Fbxw7 stable expression were subcutaneously injected into nude mice and tumor formation was monitored. The nude mice were euthanized after 26 days and the photos of the nude mice and tumors are shown. (b) Growth course of the tumors. (c) Weights of the tumors harvested from mice at the end of experiments. (d) H&E staining of the tumors in the control and Fbxw7-overexpressing groups. All the results are expressed as mean ± SD (n = 3, *∗∗* p < 0.01).

**Figure 6:** Expression of Fbxw7 and Skp2 in clinical lung adenocarcinoma tissues. (a) Immunohistochemical (IHC) staining of Fbxw7 expression in human lung adenocarcinoma tissues compared with adjacent nontumor tissues, scale bar = 50 *μ*m. (b) Comparison of the number of Fbxw7 positive cells among different tissues in IHC analysis. (c) IHC staining of Skp2 expression in human lung adenocarcinoma tissues compared with adjacent nontumor tissues, scale bar = 50 *μ*m. (d) Comparison of the number of Skp2 positive cells among different tissues in IHC analysis. All the results are expressed as mean ± SD (n = 3, *∗* p < 0.05, compared with nontumor tissues; *∗∗* p < 0.01, compared with nontumor tissues).

**Table 1:** The sequences of oligonucleotide primers.

	Primer sequences (5′ → 3′)
hGAPDH	CAATGACCCCTTCATTGACC
	GACAAGCTTCCCGTTCTCAG
Skp2	CAACTACCTCCAACACCTATCACTCA
	TGGCAATGGTGGTGAAATGG
P27	CAACTCAGCAGCGGGGTCT
	CCACGCCATCCTTGGTCTT
Fbxw7	ACGACGCCGAATTACATCTGTC
	CGTTGAAACTGGGGTTCTATCACT
c-Myc	ACATCCTGTCCGTCCAAGCA
	CACAAGAGTTCCGTAGCTGTTCAA
Oct3/4	AAGGGCAAGCGATCAAGCA
	CAGAGTGGTGACGGAGACAGG

## Data Availability

The data used to support the findings of this study are available from the corresponding author upon request.
